# m6A-Related lncRNAs Predict Overall Survival of Patients and Regulate the Tumor Immune Microenvironment in Osteosarcoma

**DOI:** 10.1155/2022/9315283

**Published:** 2022-08-08

**Authors:** Yikang Bi, Depeng Meng, Ma Wan, Ning Xu, Yafeng Xu, Kaixuan Yuan, Pengcheng Liu, Hao Fang, Hai Hu, Shenghui Lan

**Affiliations:** ^1^Department of Orthopaedics, The Eighth People's Hospital, Jiangsu University, Shanghai 200235, China; ^2^Department of Orthopaedics, Xuhui Branch of The Sixth People's Hospital, Shanghai Jiao Tong University, Shanghai 200233, China; ^3^Department of Orthopedics, Changzheng Hospital, Naval Military Medical University, Shanghai 200074, China

## Abstract

**Background:**

m6A-related lncRNAs have demonstrated great potential tumor diagnostic and therapeutic targets. The goal of this work was to find m6A-regulated lncRNAs in osteosarcoma patients.

**Method:**

The Cancer Genome Atlas (TCGA) database was used to retrieve RNA sequencing and medical information from osteosarcoma sufferers. The Pearson's correlation test was used to identify the m6A-related lncRNAs. A risk model was built using univariate and multivariable Cox regression analysis. Kaplan–Meier survival analysis and receiver functional requirements were used to assess the risk model's performance (ROC). By using the CIBERSORT method, the associations between the relative risks and different immune cell infiltration were investigated. Lastly, the bioactivities of high-risk and low-risk subgroups were investigated using Gene Set Enrichment Analysis (GSEA).

**Result:**

A total of 531 m6A-related lncRNAs were obtained from TCGA. Seven lncRNAs have demonstrated prognostic values. A total of 88 OS patients were separated into cluster 1, cluster 2, and cluster 3. The overall survival rate of OS patients in cluster 3 was more favorable than that of those in cluster 1 and cluster 2. The average Stromal score was much higher in cluster 1 than in cluster 2 and cluster 3 (*P* < 0.05). The expression levels of lncRNAs used in the construction of the risk prediction model in the high-risk group were generally lower than those in the low-risk group. Analysis of patient survival indicated that the survival of the low-risk group was higher than that of the high-risk group (*P* < 0.0001) and the area under the curve (AUC) of the ROC curve was 0.719. Using the CIBERSORT algorithm, the results revealed that Macrophages M0, Macrophages M2, and T cells CD4 memory resting accounted for a large proportion of immune cell infiltration. By GSEA analysis, our results implied that the high-risk group was mainly involved in unfolded protein response, DNA repair signaling, and epithelial-mesenchymal transition signaling pathway and glycolysis pathway; meanwhile, the low-risk group was mainly involved in estrogen response early and KRAS signaling pathway.

**Conclusion:**

Our investigation showed that m6A-related lncRNAs remained tightly connected to the immunological microenvironment of osteosarcoma tumors, potentially influencing carcinogenesis and development. The immune microenvironment and immune-related biochemical pathways can be changed by regulating the transcription of M6A modulators or lncRNAs. In addition, we looked for risk-related signaling of m6A-related lncRNAs in osteosarcomas and built and validated the risk prediction system. The findings of our current analysis will facilitate the assessment of outcomes and the development of immunotherapies for sufferers of osteosarcomas.

## 1. Introduction

Osteosarcoma (also known as osteogenic sarcoma or simply bone cancer) is the most frequent kind of bone cancer [1]. It is a type of invasive malignant neoplasm that develops from primitive altered cells of mesenchymal origin (and hence is a sarcoma) and demonstrates osteoblastic differentiating and creates cancerous osteoid [1]. The most frequent histological kind of primary bone sarcoma is osteosarcoma [2]. It is particularly common among adolescents and young adults [3]. Despite the positive results of comprehensive surgical resection along with chemotherapy and radiotherapy, roughly 40–50 percent of patients develop lung dissemination [4]. Patients with lung metastatic tumors had a five-year life expectancy of only 28% [5]. Therefore, searching for new treatment targets and prognostic biomarkers is critical.

N6-methyladenosine (m6A) is the methylated adenosine that occurs at the N6 site and it is prevalently an epigenetic alteration in mRNA and noncoding RNAs (ncRNAs) [6]. The process of m6A is considered to be dynamic and reversible. Similar to other epigenetic regulatory mechanisms, the bioactivities of m6A are coordinated by “writer,” “reader,” and “eraser” [7]. The compound of m6A-writer acts as a methylase, allowing m6A to be installed. The m6A alteration is then identified by m6A-associated proteins, which are also called as readers. The erasers are demethylases that are in charge of eliminating the m6A alterations. Several investigations have shown that m6A alterations control carcinogenesis and progression [8]. The relevance of m6A variations in malignancy prediction is becoming clear.

Long noncoding RNA (lncRNA) is RNA with a transcriptome sequence of more than 200 nucleotides that are not transcribed into proteins [9]. lncRNA is involved in a number of physiological systems in cells, including cell growth and differentiation [10]. lncRNA influences gene transcriptions at three different sides: epigenetic regulation, transcription, and posttranscription. The abnormal pattern of lncRNA is linked to cancerous aggressiveness as well. Recent evidence has proved that lncRNA acts as tumorigenesis or repressors by participating in numerous signaling pathways [11]. For instance, SRY-box transcription factor 2 (SOX2) promotes development in colorectal cancer (CRC) by catalyzing methyl with methyltransferase-like protein 3 (METTL3) [12], whereas BCL2 interacting protein 3 (BNIP3) promotes cancer progression in breast cancer by catalyzing demethylation with FTO (fat mass and obesity-associated protein) [13]. Furthermore, lncRNAs have the potential to be used as prognosis markers in various types of tumors, such as prostate, breast, and liver cancers [14]. Recently, there has been a growing interest in the research framework between m6A and lncRNAs. Their regulating complex is implicated in tumor growth, migration, and metastasis in a variety of malignancies, giving new targets for cancer diagnostics and treatment. lncRNAs and m6A have been shown to have critical roles in controlling cancer bioactivity, but the mutual regulation mechanism between them is unknown. As a result, it is critical to investigate the possible biochemical reaction of these unregulated m6A-related lncRNAs in osteosarcoma. Therefore, determining the associations between the alterations of m6A-related lncRNAs and the courses of osteosarcoma may help to find biomarkers that can be considered predictive and prognostic markers.

## 2. Materials and Methods

### 2.1. The Process of Data Acquisition

The raw data and corresponding clinical information were downloaded from Genomic Data Commons of the TCGA database(https://xenabrowser.net/datapages/?cohort=GDC%20TARGET-OS&removeHub=https%3A%2F%2Fxena.treehouse.gi.ucsc.edu%3A443). These data contained three files of clinical data (TARGET-OS.clinical.tsv.gz), expression profiles (TARGET-OS.htseq_counts.tsv.gz), and survival information (TARGET-OS.survival.tsv). Clinical data of OS patients did not include normal controls; however, the data contained a variety of other clinical information (such as metastases, tumor grade, age, and gender). According to previous studies, these cases were grouped into two groups: metastases and nonmetastases, and the sample size was balanced between the two groups [15]. The available literature yielded a total of 20 m6A regulatory factors, including WTAP, METTL3, METTL14, METTL16, KIAA1429, ZC3H13, RBM15, HNRNPA2B1, IGF2BP1, IGF2BP2, IGF2BP3, YTHDC1, YTHDC2, FMR1, LRPPRC, YTHDF1, YTHDF2, YTHDF3, ALKBH5, and FTO.

### 2.2. Screening of Prognostic Genes

In accordance with the TCGA naming convention, all samples ending in 01A were OS samples, including 88 cases in total in our study. Gene IDs for TCGA-OS expression profiles were converted using the package (org.Hs.eg.db), obtaining a total of 34446 gene symbols. When there was a single symbol corresponding to multiple IDs, the expression profiles of identical gene symbols were merged by the maximum value. The GRCh38 annotation file was downloaded from the GENCODE website, which was used to differentiate the types of genes for TCGA-STAD expression profiles. The expression profiles of 20 m6A-related genes were extracted and box-line plots were plotted using the ggplot2 package. Correlation analysis was conducted on the expression profiles of all samples using the rcorr function of the Hmisc package. The correlation cor values and *p* values of the 10 m6A-related genes with lncRNA genes were obtained using Pearson analysis (*p* value < 0.05, cor Filter>0.2) [16]. A total of 531 m6A-related lncRNAs were obtained.

### 2.3. Cox Regression Analysis

Clinical data packages for survival time and survival status were combined with 531 lncRNA gene expression profiles associated with m6A. One-way Cox regression analysis was performed using the R package survivor (*p* value < 0.05). Correlation analysis was carried out using the cor.test of the stats package (*p* value < 0.05).

### 2.4. Consistent Clustering Analysis

The expression profiles of seven lncRNA prognostic genes associated with disease risk were analyzed by consistent clustering using the R package consensus cluster plus, setting the number of clusters to 2.

### 2.5. Prognosis and the Immune Microenvironment in Coherent Clustering

The expression profiles of 9 prognostic genes were mapped using the pheatmap package, plus additional grouping tags (such as age and gender), and divided into Cluster 1, Cluster 2, and Cluster 3. Survival curve analysis was performed with the survfit of the surv. package and plotted with the ggsurvplot function of the survminer package, grouped as Cluster1, Cluster2, and Cluster3. Using the CIBERSORT algorithm, immune infiltration of patient tissue is identified by 22 different types of immune cells. LM22 feature matrix file with CIBERSORT algorithm (1000 permutations) was applied to compare the immunocyte infiltration scores of Cluster1, Cluster2, and Cluster3.

Using the ESTIMATE package, immune scoring was calculated for TCGA-OS expression profiles, including ESTIMATE score, Immune score, Stromal score, and Tumor Purity. The box plots were drawn using the ggplot2 package, grouped as Cluster1, Cluster2, and Cluster3. The significance of differences between groups was calculated by *T* test.

### 2.6. Constructing the Prognosis Diagnosis Model of TCGA-OS

Risk scores were calculated for the seven lncRNAs screened that were associated with OS risks. The calculation formula is as follows:

(1) $$\begin{array}{c} \text{Risk score}=\text{coef}\left(\text{lncRNAn}\right)\times \text{expr }\left(\text{lncRNAn}\right), \end{array}$$

where coef(lncRNAn) represents the regression coefficient of lncRNA.

Based on this formula, the risk score of each group could be derived [17]. The median risk score was used to classify the OS samples containing survival information into a high-risk group and a low-risk group. The risk score distribution of the sample was plotted using the ggplot2 package. The samples were divided into high-risk and low-risk groups. The survival curves were analyzed using the survfit function of the survivor package and plotted using the ggsurvplot function of the survminer package.

### 2.7. Immune Infiltration Analysis

The LM22 feature matrix file with the CIBERSORT algorithm (1000 permutations) was used to compare the immunocyte infiltration scores of the high-risk group and low-risk group. The risk core risk scores of Cluster1, Cluster2, and Cluster3 were compared, and differences between groups were calculated using a *t*-test. The box plot was obtained by using the ggplot2 package.

### 2.8. Correlation of Immune Infiltration with lncRNA

The correlation between hub gene expression and immune infiltrating cells was calculated by the cor.test function of the psych package (spearman algorithm). Heatmaps were drawn with the pheatmap package to show the correlation heatmaps (^∗∗∗^*P* < 0.001, ^∗∗^*P* < 0.01, and ^*∗*^*P* < 0.05). The colors from blue to red indicate a correlation cor-value from small to large.

### 2.9. Gene Set Enrichment Analysis (GSEA)

GSEA analysis was performed using GSEA v4.2.2. Hallmarks (h.all.v7.5.1.symbols.gmt) were used to identify and illustrate specific signaling pathways.

## 3. Results

### 3.1. The m6A-Related Differential Genes and Identification of m6A-Related lncRNAs in OS

88 samples of OS were derived from the TCGA database. The samples were divided into two subgroups: metastases (22 specimens) and nonmetastases (65 specimens). 3039 lncRNAs and 19135 mRNAs were obtained in total. 17,249 differential genes were found using the Limma package differential analysis (*p* value < 0.05). These differential genes were intersected with 20 m6A-related genes to obtain 10 m6A-related differential genes. These ten m6A-related differential genes included WTAP, METTL14, RBM15, IGF2BP1, IGF2BP2, IGF2BP3, YTHDC2, YTHDF2, YTHDF3, and FTO.

28 lncRNA prognostic genes associated with the risk of OS were found in total. Multifactor Cox regression analysis was continued for 28 lncRNAs obtained by single-factor regression using the R package SURVIVAL (*p* value < 0.05) [17]. A total of 7 lncRNA prognostic genes were screened for association with prognostic significance (Table 1). The expression profiles of 10 differential genes regulated by m6A and 7 lncRNA prognostic genes associated with risk factors were extracted separately. The correlation between m6A-related genes and lncRNAs is shown in Figure 1.

### 3.2. Consensus Clustering Categorized OS Patients according to m6A-Related Prognostic lncRNAs

Following the transcription of m6A-related predictive lncRNAs, consensus clustering was also used to divide OS patients into different clusters (Figure 2). Due to the similarities demonstrated by the expression profiles of m6A-related predictive lncRNAs, *k* = 3 was discovered to be the best clustering consistency from *k* = 2 to 9 (Figure 2(a)). A total of 88 OS patients were separated into cluster 1, cluster 2, and cluster 3. The overall survival rate of OS patients in cluster 3 was more favorable than that of those in cluster 1 and cluster 2 (Figure 2(b), *p* = 0.00081).

### 3.3. Consensus Clustering Linked to Immune Infiltration

To explore the role of m6A-related prognostic lncRNAs in the osteosarcoma immune microenvironment, we then analyzed the difference in the immune score and immune cell infiltration level among cluster 1, cluster 2, and cluster 3. The average Stromal score was much higher in cluster 1 than those in cluster 2 and cluster 3 (Figure 3) (*P* < 0.05).

### 3.4. Risk Signaling of m6A-Related lncRNAs and Risk Prediction Model Showed Prognostic Value in Osteosarcoma

After calculating the risk scores of individual patients, the cases were divided into a high-risk group and a low-risk group based on the median risk score (Figure 4(a)). The heatmap showed changes in the risk score and expression levels of lncRNAs. The expression levels of lncRNAs used in the construction of the risk prediction model in the high-risk group were generally lower than those in the low-risk group (Figure 4(e)). Analysis of patient survival indicated that the survival of the low-risk group was higher than that of the high-risk group (*P* < 0.0001, Figure 4(d)). The area under the curve (AUC) of the ROC curve was 0.719, indicating that the model showed medium accuracy in predicting the prognosis of osteosarcoma patients (Figure 4(e)). Our results showed that m6A-related lncRNAs had prognostic value and that the risk prediction model showed satisfactory performance in predicting the prognosis of patients with osteosarcoma (Figure 4).

### 3.5. Correlations between Immune Infiltration and m6A-Related lncRNAs in Osteosarcoma

The infiltration of 22 immune cell types in osteosarcoma samples was further analyzed using the CIBERSORT algorithm. The results revealed that Macrophages M0, Macrophages M2, and T cells CD4 memory resting accounted for a large proportion of immune cell infiltration (Figure 5). However, there were no significant differences in the proportion of most of the infiltrated immune cell types between the high- and low-risk groups. The correlation coefficients between 22 types of immune cells are depicted in Table 2 and Figure 6.

### 3.6. The m6A-Related lncRNAs Subgroups Were Associated with Biological Characteristics of Osteosarcoma

Next, we analyzed differences in the biological responses of the subgroups generated using consensus clustering in order to further explore the relationships between m6A-related lncRNAs clustering subgroups and osteosarcoma biological characteristics. GSEA was used to explore the main KEGG signaling pathways in the two subgroups. Our results showed that the high-risk group was mainly involved in unfolded protein response, DNA repair signaling, and epithelial-mesenchymal transition signaling pathway and glycolysis pathway (Figures 7(a)–7(d)), which are related to the initiation of metastasis in cancer progression [18–20]. The low-risk group was mainly involved in estrogen response early and KRAS signaling pathway (Figures 7(e) and 7(f)), which are important for oncogene of osteosarcoma [21, 22]. These results indicated that there were differences in biological characteristics between high-risk and low-risk groups, which affected tumorigenesis and progression of osteosarcoma and survival of osteosarcoma patients.

## 4. Discussion

With the advancement of high-throughput sequencing methods and their widespread use in oncology, disclosing epigenomic irregularities during tumor onset and progression opens the door to the proof of identity of targeted therapies and predictive biomarkers in a range of tumors [23]. Current attention has been focused on the comprehensive detection of high sequencing results using publicly available databases, which has resulted in several major findings in the diagnosis and therapy of malignancies [17, 24]. Conversely, the involvement of m6A regulators in lncRNA deregulation in human cancer is unknown. Few research studies investigated the associations between m6A alterations and lncRNA-dependent osteosarcoma.

To elucidate the underlying biological mechanisms of the m6A-related lncRNA profile, we identified genes that were expressed differently between the metastases and nonmetastases groups. A total of 7 lncRNA prognostic genes were screened for association with prognostic significance in osteosarcoma patients (including TNS1-AS1, WWC2-AS1, TFPI2-DT, LINC01474, LINC00910, LINC01982, and LINC00538). We did a clustering analysis based on the transcriptome of m6A-related predictive lncRNAs to further investigate the association between m6A-related lncRNAs and the clinical and pathological and biological aspects of AML. This analysis produced three subgroups, which were labeled as cluster 1, cluster 2, and cluster 3. The overall survival rate of OS patients in cluster 3 was more favorable than that of those in cluster 1 and cluster 2.

In addition, the samples were separated into two groups according to the average risk score: high-risk and low-risk groups after computing the risk scores of patient characteristics. GSEA suggested that the high-risk group was mostly engaged in unfolded protein response, DNA repair signaling, epithelial-mesenchymal transition signaling, and glycolysis signaling pathways. The low-risk group was mainly involved in estrogen response early and KRAS signaling pathway. The low-risk group had a better overall survival rate than the high-risk group did. The ROC curve's area under the curve (AUC) was 0.719, meaning that the model was somewhat capable of predicting the prognosis of osteosarcoma patients. According to a prior study, the active unfolded protein response was a key biochemical characteristic of osteosarcoma [25]. A large amount of evidence about the involvement of DNA damage response in osteosarcoma formation, survival, and treatments was assembled in a review paper [26].

Diverse immune cells and released substances make up the immunological microenvironment [27]. Tumor cell invasion, immunological capabilities, and the activation of targeted therapies could all determine cancer patients' outcomes and forecast their responsiveness to immunotherapies [28, 29]. The immunological microenvironment and immune-related biochemical pathways could be altered by modulating the transcription of m6A regulatory or lncRNAs [30]. Our results revealed that Macrophages M0, Macrophages M2, and T cells CD4 memory resting accounted for a large proportion of immune cell infiltration. It is reported that M2 macrophages can encourage tumor progression [31, 32]. Especially, elevated infiltration of M2 macrophages has been linked to osteosarcoma metastases and poor patient outcomes, notwithstanding the adoption of intensive therapy regimens [33]. Moreover, exosomes from metastasis osteosarcoma cells have been shown to alter tumor-associated macrophage cellular signaling, boost the M2 phenotype, and establish an immunosuppressive, tumor-promoting milieu via producing TGFB2 [34]. However, there were no significant differences in the proportion of most of the infiltrated immune cell types between the high- and low-risk groups.

We investigated the association between m6A-related lncRNAs expression and the levels of immune infiltration in OS using CIBERSORT. TNS1-AS1 and TFPI2-DT were found positively correlated with B cell memory and B cells naive in our data, respectively. These results about immune infiltrate in osteosarcomas were consistent with previous studies [35, 36]. Additionally, the results uncovered that LINC01474 had a positive correlation with T cells CD8; however, LINC00910 was negatively related to T cells CD8. Other scholars believed that the significant infiltration of T cells CD8 activation in tumors may aid our signature's capacity to attain consistent predictive value [37]. There has been proof that programmed death-1 receptor (PD-1) plays a role in the evolution of osteosarcomas, and the proportion of PD-1 in blood CD8+ T cells is much higher in osteosarcomas patients [38, 39]. Moreover, LINC00538 was positively correlated with dendritic cells resting, in the meanwhile, negatively linked to dendritic cells activated in our results. Previous studies demonstrated that the proportions of dendritic cells resting were positively correlated with the risk score of osteosarcomas [40] and LINC00538 was highly associated with worse outcomes of colon cancer patients [41].

There are some disadvantages to our study as well. First, for starters, the study's findings need to be verified by bigger external partners. Second, more specific methods of interaction between m6A and lncRNAs, as well as how this regulation pattern contributes to the reshaping of TME, should be investigated further. Third, it should be examined if m6A-related lncRNAs participate in other biological processes associated with cancer. Lastly, while the associations between the risk score and histopathological characteristics or TME had a significant difference, the medical variations should be confirmed again because the variance was not as apparent. To validate the prediction models built in our current investigation, additional research studies should incorporate specimens from other databases as well as an increasing number of clinical specimens. More research is needed to completely understand the signaling pathways of m6A-related lncRNAs in the carcinogenesis and development of osteosarcomas. This study has some limitations: although the results of this study have some innovative and clinical significance, they have not been verified by more evidence, which makes this study incomplete, and a confirmatory study will be added in the future to make up for the shortcomings of this study.

In conclusion, our investigation showed that m6A-related lncRNAs remained tightly connected to the immunological microenvironment of osteosarcoma tumors, potentially influencing carcinogenesis and development. In addition, we looked for risk-related signaling of m6A-related lncRNAs in osteosarcomas and built and validated the risk prediction system. The findings of our current analysis will facilitate the assessment of the outcome and the development of immunotherapies for sufferers of osteosarcomas.

## Figures and Tables

**Figure 1:** The correlation between 10 m6A-related genes and 7 lncRNA prognostic genes. ^*∗*^*P* < 0.05; ^∗∗^*P* < 0.01.

**Figure 2:** Consensus clustering of m6A-related prognostic lncRNAs. (a) TCGA osteosarcoma cohorts were grouped into three clusters according to the consensus clustering matrix (*k* = 3). (b) Overall survival analysis revealed a better overall survival of osteosarcoma patients in cluster 3 than those in cluster 1 and cluster 2. (c) The heatmap of the 3 clusters along with general information of patients.

**Figure 3:** (a) The comparison of the immune score between the low-risk and high-risk groups (*p* > 0.05). (b–e) Comparison of immune score: (b) Stromal score, (c) Immune score, (d) ESTIMATE Score, and (e) Tumor Purity.

**Figure 4:** (a) The risk score distribution; (b) survival time scatter diagram; (c) clinical and pathological characteristics and varied lncRNA expression patterns in high- and low groups are depicted in a heatmap; (d) the risks model's Kaplan–Meier survival line; (e) ROC curve analysis.

**Figure 5:** The violin plot of 22 tumor-infiltrating immune cell types in low- and high-risk groups. The infiltration of 22 immune cell types in osteosarcoma was analyzed by the CIBERSORT algorithm.

**Figure 6:** The correlations between immune infiltration and m6A-related lncRNAs. ^*∗*^*P* < 0.05; ^∗∗^*P* < 0.01.

**Figure 7:** Abnormally activated signaling pathways in the two subgroups after Gene Set Enrichment Analysis. (a–d) Performed in the high-risk group, including unfolded protein response (ES = 0.42, *P*=0.02, FDR = 0.110), DNA repair signaling pathway (ES = 0.41, *P*=0.0096, FDR = 0.070), epithelial-mesenchymal transition signaling pathway (ES = 0.55, *P*=0.032, FDR = 0.337), and glycolysis pathway (ES = 0.44, *P*=0.032, FDR = 0.087). (e–f) Performed in the low-risk group, including estrogen response early (ES = 0.40, *P*=0.038, FDR = 1.0) and KRAS signaling pathway (ES = 0.40, *P*=0.039, FDR = 1.0).

**Table 1:** Seven m6A-related lncRNAs with prognostic significance in osteosarcoma identified by Cox regression analysis.

lncRNA	Coefficient	HR (95% CI)	HR95%L	HR95%H	*p*
TNS1-AS1	−0.978	0.376 (0.191–0.74)	0.191	0.74	0.005
WWC2-AS1	1.095	2.989 (1.319–6.775)	1.319	6.775	0.009
TFPI2-DT	−1.124	0.325 (0.141–0.748)	0.141	0.748	0.008
LINC01474	−1.756	0.173 (0.049–0.609)	0.049	0.609	0.006
LINC00910	5.869	354.031 (3.782–33142.623)	3.782	33142.623	0.011
LINC01982	−0.972	0.378 (0.146–0.98)	0.146	0.98	0.045
LINC00538	1.201	3.324 (1.158–9.539)	1.158	9.539	0.026

**Table 2:** The correlations between immune infiltration and m6A-related lncRNAs.

lncRNA	Immune process	Positive (+)/negative (–) correlation	*r*	*P* value
TNS1-AS1	B cell memory	**+**	0.21	0.048
TFPI2-DT	B cells naive	**+**	0.23	0.034
LINC01474	T cells CD8	**+**	0.25	0.020
LINC01474	T cells CD4 memory activated	**+**		0.009
LINC00910	T cells CD8	–	−0.21	0.049
LINC00538	T cells CD4 naive	**+**	0.34	0.001
LINC00538	Dendritic cells resting	**+**	0.25	0.017
LINC00538	Dendritic cells activated	–	−0.23	0.035

## Data Availability

The datasets used and analyzed during the current study are available from the corresponding author upon reasonable request.

## References

[1] Luetke A., Meyers P. A., Lewis I., Juergens H. (2014). Osteosarcoma treatment - where do we stand? A state of the art review. *Cancer Treatment Reviews*.

[2] Ottaviani G., Jaffe N. (2009). The epidemiology of osteosarcoma. *Cancer Treatment and Research*.

[3] Wang S., Zhong L., Li Y. (2019). Up-regulation of PCOLCE by TWIST1 promotes metastasis in Osteosarcoma. *Theranostics*.

[4] Hirahata M., Osaki M., Kanda Y. (2016). PAI ‐1, a target gene of miR‐143, regulates invasion and metastasis by upregulating MMP ‐13 expression of human osteosarcoma. *Cancer Medicine*.

[5] Yu X., Hu L., Li S. Y. (2019). Long non-coding RNA Taurine upregulated gene 1 promotes osteosarcoma cell metastasis by mediating HIF-1*α* via miR-143-5p. *Cell Death & Disease*.

[6] He L., Li H., Wu A., Peng Y., Shu G., Yin G. (2019). Functions of N6-methyladenosine and its role in cancer. *Molecular Cancer*.

[7] Meyer K. D., Jaffrey S. R. (2017). Rethinking m6A readers, writers, and erasers. *Annual Review of Cell and Developmental Biology*.

[8] Wang T., Kong S., Tao M., Ju S. (2020). The potential role of RNA N6-methyladenosine in Cancer progression. *Molecular Cancer*.

[9] Chen Y., Li Z., Chen X., Zhang S. (2021). Long non-coding RNAs: from disease code to drug role. *Acta Pharmaceutica Sinica B*.

[10] Wang W., Min L., Qiu X. (2021). Biological function of long non-coding RNA (LncRNA) xist. *Frontiers in Cell and Developmental Biology*.

[11] Huarte M. (2015). The emerging role of lncRNAs in cancer. *Nature Medicine*.

[12] Li T., Hu P. S., Zuo Z. (2019 Jun 24). METTL3 facilitates tumor progression via an m6A-IGF2BP2-dependent mechanism in colorectal carcinoma. *Molecular Cancer*.

[13] Niu Y., Lin Z., Wan A. (2019). RNA N6-methyladenosine demethylase FTO promotes breast tumor progression through inhibiting BNIP3. *Molecular Cancer*.

[14] Qian Y., Shi L., Luo Z. (2020). Long non-coding RNAs in cancer: implications for diagnosis, prognosis, and therapy. *Frontiers of Medicine*.

[15] Tian H., Guan D., Li J. (2018). Identifying osteosarcoma metastasis associated genes by weighted gene co-expression network analysis (WGCNA). *Medicine*.

[16] Yuan H., Liu J., Zhao L. (2021). Prognostic risk model and tumor immune environment modulation of m5C-related LncRNAs in pancreatic ductal adenocarcinoma. *Frontiers in Immunology*.

[17] Pan J., Huang Z., Xu Y. (2021). m5C-Related lncRNAs predict overall survival of patients and regulate the tumor immune microenvironment in lung adenocarcinoma. *Frontiers in Cell and Developmental Biology*.

[18] Wang G., Fan Y., Cao P., Tan K. (2022). Insight into the mitochondrial unfolded protein response and cancer: opportunities and challenges. *Cell & Bioscience*.

[19] Lagunas A. M., Wu J., Crowe D. L. (2017). Telomere DNA damage signaling regulates cancer stem cell evolution, epithelial mesenchymal transition, and metastasis. *Oncotarget*.

[20] Gonzalez D. M., Medici D. (2014). Signaling mechanisms of the epithelial-mesenchymal transition. *Science Signaling*.

[21] Traphagen N. A., Hosford S. R., Jiang A. (2021). High estrogen receptor alpha activation confers resistance to estrogen deprivation and is required for therapeutic response to estrogen in breast cancer. *Oncogene*.

[22] Kim H. J., Lee H. N., Jeong M. S., Jang S. B. (2021). Oncogenic KRAS: signaling and drug resistance. *Cancers*.

[23] Zhao J., Dean D. C., Hornicek F. J., Yu X., Duan Z. (2020). Emerging next-generation sequencing-based discoveries for targeted osteosarcoma therapy. *Cancer Letters*.

[24] Zhong F., Yao F., Cheng Y. (2022). m6A-related lncRNAs predict prognosis and indicate immune microenvironment in acute myeloid leukemia. *Scientific Reports*.

[25] Shi C., Zhao F., Zhang T. (2022). A novel prognostic signature in osteosarcoma characterised from the perspective of unfolded protein response. *Clinical and Translational Medicine*.

[26] Sadoughi F., Maleki Dana P., Asemi Z., Yousefi B. (2021). DNA damage response and repair in osteosarcoma: defects, regulation and therapeutic implications. *DNA Repair*.

[27] Hayase E., Jenq R. R. (2021). Role of the intestinal microbiome and microbial-derived metabolites in immune checkpoint blockade immunotherapy of cancer. *Genome Medicine*.

[28] Price G., Bouras A., Hambardzumyan D., Hadjipanayis C. G. (2021). Current knowledge on the immune microenvironment and emerging immunotherapies in diffuse midline glioma. *EBioMedicine*.

[29] Zhang K., Ping L., Du T. (2021). A ferroptosis-related lncRNAs signature predicts prognosis and immune microenvironment for breast cancer. *Frontiers in Molecular Biosciences*.

[30] Xu F., Huang X., Li Y., Chen Y., Lin L. (2021). m6A-related lncRNAs are potential biomarkers for predicting prognoses and immune responses in patients with LUAD. *Molecular Therapy - Nucleic Acids*.

[31] Fu X., Shi H., Qi Y., Zhang W., Dong P. (2015). M2 polarized macrophages induced by CSE promote proliferation, migration, and invasion of alveolar basal epithelial cells. *International Immunopharmacology*.

[32] Schmieder A., Michel J., Schönhaar K., Goerdt S., Schledzewski K. (2012). Differentiation and gene expression profile of tumor-associated macrophages. *Seminars in Cancer Biology*.

[33] Cersosimo F., Lonardi S., Bernardini G. (2020). Tumor-associated macrophages in osteosarcoma: from mechanisms to therapy. *International Journal of Molecular Sciences*.

[34] Wolf-Dennen K., Gordon N., Kleinerman E. S. (2020). Exosomal communication by metastatic osteosarcoma cells modulates alveolar macrophages to an M2 tumor-promoting phenotype and inhibits tumoricidal functions. *OncoImmunology*.

[35] Huang H., Tan M., Zheng L. (2021). Prognostic implications of the complement protein C1Q and its correlation with immune Infiltrates in osteosarcoma. *OncoTargets and Therapy*.

[36] Sun J., Xu H., Qi M., Zhang C., Shi J. (2019). Identification of key genes in osteosarcoma by meta‑analysis of gene expression microarray. *Molecular Medicine Reports*.

[37] Yang J., Zhang A., Luo H., Ma C. (2022). Construction and validation of a novel gene signature for predicting the prognosis of osteosarcoma. *Scientific Reports*.

[38] Wang Z., Li B., Ren Y., Ye Z. (2016). T-Cell-Based immunotherapy for osteosarcoma: challenges and opportunities. *Frontiers in Immunology*.

[39] Farhood B., Najafi M., Mortezaee K. (2019). CD8 + cytotoxic T lymphocytes in cancer immunotherapy: a review. *Journal of Cellular Physiology*.

[40] Zhang C., Zheng J. H., Lin Z. H. (2020). Profiles of immune cell infiltration and immune-related genes in the tumor microenvironment of osteosarcoma. *Aging*.

[41] Tang H., Dou Y., Meng Y., Lu Q., Liang L., Luo Y. (2020). LINC00538 promotes the progression of colon cancer through inhibiting NKD2 expression. *J BUON*.

